# 2D-convolutional neural network based fault detection and classification of transmission lines using scalogram images

**DOI:** 10.1016/j.heliyon.2024.e38947

**Published:** 2024-10-04

**Authors:** Pravati Nayak, Shitya Ranjan Das, Ranjan K. Mallick, Sairam Mishra, Ahmed Althobaiti, Alsharef Mohammad, Flah Aymen

**Affiliations:** a Department of Electrical Engineering, Siksha ‘O’ Anushandhan deemed to be University, Bhubaneswar, Odisha, PIN-751030, India; b Department of Electrical and Electronics Engineering, Siksha ‘O’ Anushandhan deemed to be University, Bhubaneswar, Odisha, PIN-751030, India; c Electrical Engineering Department, Taif University, Saudi Arabia; d Energy Processes Environment and Electrical Systems Unit, National Engineering School of Gabes, University of Gabes, Gabes, 6029, Tunisia; e MEU Research Unit, Middle East University, Amman, 11831, Jordan; f College of Engineering, University of Business and Technology (UBT), Jeddah, 21448, Saudi Arabia; g Private Higher School of Applied Sciences and Technology of Gabes, University of Gabes, Gabes, 6029, Tunisia; h Applied Science Research Center, Applied Science Private University, Amman, 11931, Jordan; i ENET Centre, VSB-Technical University of Ostrava, Ostrava, Czech Republic

**Keywords:** Fault detection, Wavelet transform, Convolutional neural networks, Transmission lines

## Abstract

The reliable operation of power transmission systems is essential for maintaining the stability and efficiency of the electrical grid. Rapid and accurate detection of faults in transmission lines is crucial for minimizing downtime and preventing cascading failures. This research presents a novel approach to fault detection and classification in transmission lines employing 2D Convolutional Neural Networks (2D-CNN).The proposed methodology leverages the inherent spatial characteristics of fault signals, converting them as 2D scalogram images for input to the CNN model. By converting fault signals into scalogram representations, the network can capture both temporal and frequency domain features, enabling a more comprehensive analysis of fault patterns. The 2D-CNN architecture is designed to automatically learn hierarchical features, allowing for effective discrimination between different fault types. To evaluate the performance of the proposed approach, extensive simulations and experiments were conducted using MATLAB/SIMULINK modeled transmission line data. The results demonstrate the superior fault detection accuracy and classification capabilities of the 2D-CNN model. The performance of the proposed model is evaluated using 10-fold cross-validation, and its effectiveness is assessed by comparing it with current state-of-the-art techniques. Proposed 2D-CNN model has evidenced an accuracy of 99.9074 with ideal dataset for 12- class fault classification and performing consistently in presence of noise, having an accuracy of 99.629 %,99.72 % and 99.814 % in 20.30 and 40 dB noises respectively. The proposed model also verified in high resistance fault condition. The model exhibits robustness to noise and is capable of generalizing well to various fault scenarios. The proposed methodology offers a scalable and efficient solution for transmission line fault analysis, paving the way for the integration of advanced machine learning techniques into the operation and maintenance of power transmission infrastructure.

**Table:** Abbreviation/Acronym/Symbol

Abbreviation/Acronym/Symbol	Interpretation
2D	Two dimensional
1D	One dimensional
2D-CNN	2D Convolutional Neural Networks
NN	Neural Networks
SVM	Support Vector Machines
DT	Decision Trees
SVM	Support Vector Machines
DWT	Discrete wavelet transform
CWT	continuous wavelet transform
RFC	Random Forest classifiers
LSTM	Long Short-Term Memory
HHT	Hilbert-Hang Transform
PNN	probabilistic neural network
ELM	Extreme learning Machine
RGB	"Red, Green, Blue."
t-SNE	t-Distributed Stochastic Neighbor Embedding.
SNR	signals to noise ratio
LG	Line to ground
LLG	Double line to ground
LLLG	Triple line to ground
HRF	High resistance fault

## 1 Introduction

The reliable operation of power transmission systems is a foundation for the stability and efficiency of electrical grids worldwide. Transmission lines, being the backbone of electrical networks, are always exposed to various faults such as short circuits, open circuits, and grounding issues. These faults can lead to severe disruptions, including power outages and potential damage to infrastructure, affecting both utilities and consumers. Therefore, the rapid and accurate detection and classification of faults in transmission lines are of paramount importance to ensure continuous and reliable power delivery.

### 1.1 Motivation and Incitement

Traditional methods for fault detection and classification, such as impedance-based techniques and traveling wave methods, while effective, often suffer from limitations in terms of speed, accuracy, and adaptability to different fault conditions. With the increasing complexity and scale of modern power systems, there is a pressing need for more advanced and robust fault analysis techniques.

Recent advancements in machine learning, particularly in the field of deep learning, offer promising solutions to these challenges. Convolutional Neural Networks (CNNs), a class of deep learning models, have demonstrated exceptional performance in various image recognition and classification tasks due to their ability to automatically learn and extract hierarchical features from data. This capability can be leveraged for fault detection and classification in transmission lines by transforming fault signals into a form that CNNs can effectively process.

### 1.2 Literature review

Disturbances within transmission lines pose a significantly higher risk of faults compared to other electrical components [1]. Literature suggests that approximately 80 % of electric service interruptions stem from failures within the delivery network [2]. Various types of faults, including those occurring across multiple phases simultaneously, single phases, or between phases and ground, challenge the integrity of transmission lines. To mitigate these risks, protective devices such as relays are deployed to shield transmission lines [3]. These relays respond to changes in voltage and current levels by activating trip signals to separate faulty sections swiftly. Fast fault detection and identification are crucial for safeguarding the stability of the power system and minimizing adverse effects, thus necessitating fault classification techniques [4]. With the complexity of modern power networks making manual fault recognition and clearance impractical, there is an increasing need for automatic and intelligent fault clearance systems [5]. Such systems utilize intelligent fault pattern classifiers to differentiate between pre-fault and post-fault conditions, aiding in rapid fault recognition and clearance [6]. This emphasizes the prominence of developing intelligent fault checking and diagnosis systems capable of accurately locating and classifying various types of faults to maintain power system stability and prevent unnecessary electricity loss in certain regions.

Various intelligent classification techniques, including Neural Networks (NN), Support Vector Machines (SVM), Decision Trees(10.13039/100001588DT), and Random Forest classifiers(RFC), are commonly employed in problem-solving scenarios [[5], [6], [7]]. Despite containing comprehensive information, raw current and voltage signals are challenging to interpret intelligently. Feature extraction techniques are thus utilized to extract pertinent information and mitigate the impact of system variance. Employing proper feature extraction techniques enhances awareness of fault classification or location issues, enabling more coherent and efficient solutions [5]. Different Artificial Neural 10.13039/100031212Network (ANN) models find applications across numerous fields, including fault detection in transmission lines and distribution systems [6]. Support Vector Machines (SVM), a statistical learning concept employing adaptive computational methods, map input vectors nonlinearly into a high-dimensional feature space. By determining an optimal hyper-plane, SVM maximizes the fault classifier and locator's capabilities [7]. Pre-processing, including feature extraction, is a crucial step in designing a fault classifier. The exponential increase in data dimensionality demands reliability during analysis. Feature extraction and selection tasks are essential to identify key attributes for precise fault recognition, thereby alleviating computational burden and avoiding erroneous outputs [4,7].

Wavelet transform(WT) stands out as a widely utilized method for feature extraction in fault diagnosis systems. Most studies opt for discrete wavelet transform (DWT) over continuous wavelet transform (CWT) to decompose original current and voltage signals, thus revealing signal characteristics across multiple frequency bands [8]. Artificial Neural Networks (ANNs) are a class of nonlinear statistical models and learning algorithms designed to mimic the interconnected behaviour of neurons in biological systems. Over time, ANNs have evolved and gained prominence across various disciplines. Similarly, Support Vector Machines (SVMs) have garnered significant consideration from the data mining, pattern recognition, and machine learning societies due to their excellent generalization capability, optimum solutions, and discriminative power [9]. Decision trees, as basic classifiers, assess fault occurrence based on mappings between object attributes and values [10]. This hierarchical process involves disintegrating datasets into smaller subsets to facilitate tree growth. Decision trees handle both categorical and numerical data, with nodes including leaf and decision nodes, and the uppermost decision node referred to as the root node [11,12]. Random Forest classifiers(RFC) represents an collaborative learning method designed to address classification and regression challenges. Ensemble learning enhances accuracy by combining multiple models to solve a given problem. This approach, particularly beneficial for unstable classifiers, reduces variance and yields more reliable outcomes. A common ensemble technique involves majority voting, where the label assigned to an unlabeled sample is determined by the most frequently occurring label among various classifiers. Majority voting is popular due to its simplicity and effectiveness [11,12]. In a study [13], the capabilities of Support Vector Machines (SVM) and RF in image classification were compared, revealing SVM's superior accuracy. Additionally, Long Short-Term Memory (LSTM) networks were proposed in Ref. [14] for feature extraction from time series data related to fault signals, achieving an impressive 99.7 % accuracy in a two-class scenario. Furthermore, Artificial Neural Networks (ANNs) were utilized for fault classification in Ref. [15], achieving a notable accuracy of 97.7 %. Another study [16] also employed ANN-based fault classification, demonstrating an accuracy of 84.40 % across three classes.

In recent years, there has been a growing interest among researchers in leveraging deep learning techniques for applications in power systems. Among these, the Convolutional Neural Network (CNN) has emerged as a popular tool. CNNs are a type of feed forward neural network capable of automatically extracting features from data using convolutional structures. Unlike traditional methods, CNNs eliminate the need for manual feature extraction. Inspired by biological visual perception, the architecture of CNNs consists of artificial neurons, with CNN kernels acting as receptors that respond to various features. Activation functions simulate the process by which neural signals exceeding a certain threshold are transmitted to subsequent neurons. Loss functions and optimizers are designed to guide the CNN system in learning the desired outcomes [17]. In Ref. [18] author proposed a deep-learning based fault classification technique for distribution systems, where energy matrix based on time-frequency is constructed using Hilbert-Hang Transform (HHT) and converted to digital image and fed to CNN as input. It is found that HHT-CNN capable of classifying faults in distribution system with higher accuracy. In Ref. [19] author proposed an ultrafast fault detection scheme combining discrete wavelet transform(DWT) and ANN, where DWT is applied to extract high frequency components of arial modal currents and probabilistic neural network(PNN) utilized for fault classification. Results shows that DWT-PNN provides precise classification using only one eighth of a cycle of post-event data. In Ref. [20] author proposed PNN for fault classification, differencing –based fault signals are used as input to PNN and author achieved classification accuracy of 99.32 % only using one-sixth of the post fault signals. An advanced machine learning approach known as summation-wavelet extreme learning machine (SWELM) is presented in Ref. [21] that integrates feature extraction in learning process and achieved classification accuracy of 98.22 %. Recently author uses half of a cycle's worth of post-fault current data, which is processed using the **Maximum Overlap Discrete Wavelet Packet Transform (MODWPT)**. This helps in calculating an energy-related feature for fault detection. The method was tested on a modified version of the **Western System Coordinating Council (WSCC) 9-bus system**, which includes a **Thyristor-Controlled Series Capacitor (TCSC)** It was also tested for use with wind farms in a grid-connected setup and obtained an accuracy of 100 % [22].In article [23] Truncated Singular Value Decomposition(TSVD) is used for matrix decomposition and dataset preparation, recurrent perceptron neural network(RPNN) proposed for detecting and classifying the faults in transmission system and achieved an accuracy of 99.77 % with 20 dB noise. In Ref. [24] author proposed an unsupervised frame work for fault diagnosis of TL based on Capsule Network(CN) instead of using base CN and time series image is fed to CN. An accuracy of 98 % achieved in 10 dB noise. A CNN founded fault phase identification scheme is proposed for double circuit line in Ref. [25]. Simulation is carried out in PSCAD, in test-set-A author used 7283 images as input data and obtained an accuracy of 98.27 %, in test-set-B used 1029 images and obtained an accuracy of 98.25 % and in test-set-C used 5145 images and obtained an accuracy of 98.10 %.In Ref. [26] hybrid model of CNN and LSTM is proposed with eleven no of fault classes and achieved an accuracy of 98.60 %. Recently in Ref. [27] ELM is proposed for fault detection and classification in TL and achieved an accuracy of 99.18 %.Deep learning is successfully implemented in power system research and out performs most of the data-driven techniques employed in protection, forecasting and stability analysis [28]. In Ref. [29] the proposed technique extracts key features from current signals using Variational Mode Decomposition (VMD), which breaks the signals into components of different frequency bands efficiently. These components are then converted into grey-scale images, which are classified using a Deep Convolutional Neural Network (CNN) to detect faults. The method is tested on a wind farm system with UPFC compensation, and achieves fast fault detection with higher accuracy. In recent past, the article [30] presents a fault detection and classification (FDC) scheme for a power transmission line with TCSC compensation and a large-scale DFIG wind farm. It uses RGB images of frequency features from current signals, obtained through the SPF technique, to train and test a CNN classifier. The method is validated on different power systems (2-bus, WSCC 9-bus, and IEEE 39-bus system and demonstrates high fault detection accuracy (100 %) and classification accuracy (around 99.3%–99.5 %) across the test networks. In Ref. [31] author presents a faulted line localization technique based on CNN and bus voltage.2D- CNN is proposed by author to design client driven video summarization framework in Ref. [32]. In Ref. [33] 2D-CNN is proposed for predicting antigenic variants of virus Top of Form. In summary, the major advantage of using CNNs for fault classification in transmission lines lies in their ability to automatically learn spatial hierarchies, capture relevant features, exhibit translation invariance and effectively handle large datasets. These characteristics make CNNs well-suited for tasks where the identification of complex patterns in data is crucial, such as detecting transmission line faults.

### 1.3 Contribution and paper organization

In the proposed research, a 2D-CNN-based deep learning model is developed for the task of fault detection and classification in power transmission systems. The methodology involves creating scalogram images of faulted signals using wavelet transform, which are then utilized as input for the 2D-CNN. A significant number of simulated signals are generated to represent both fault-free conditions and various types of faults, considering diverse fault locations and resistances. The performance of the proposed model is evaluated using 10-fold cross-validation, and its effectiveness is assessed by comparing it with current state-of-the-art techniques. The main contributions of this research are as follows:

A novel 2D-CNN Deep learning model is proposed for fault diagnosis of transmission line.

i) The 1-D time amplitude of fault signals are converted to 2D-scalogram images using Continuous wavelet transform to capture the inherent features of fault signals and improve fault classification accuracy.
ii) Extensive simulation study is carried out for 11 types of transmission line faults with varying parameters of transmission line and fault resistances.
iii) Design of 2D-CNN model with appropriate hyper parameters.
iv) Finally the proposed Deep learning based 2D-CNN classifier is tested in presence of different noises.
v) The proposed model also verified in high resistance fault condition.
vi) Accuracy of proposed technique is compared with current state-of-art techniques.

The remainder of this article is structured as follows: Section 2 details the system under study for modeling transmission lines, while Section 3 introduces the basics of 2D-CNN. Section 4 delvers into continuous wavelet transform and the preparation of scalogram images. Section 5 outlines the data collection and signal processing stages, and Section 6 presents the proposed 2D-CNN technique for fault detection and classification. Section 7 investigates performance, Section 8 provides the conclusion, and Section 9outlines the future scope of the proposed research.

## 2 System under study

The simulation model of the transmission network is shown in figure-1and is carried out with the help of MATLAB SIMULINK environment [34]. The total power system model consists of three areas with generating capacities of 400 kV each, linked by 300 km long transmission lines with respect to each other and the transmission lines are of distributed model type. The signal samples of fault current in p.u. values are collected from the relaying point for different fault conditions. The parameters of transmission lines are taken as,

Z_L0_ = 96.45+j335.26 Ω (Zero sequence impedance)

Z_L1_ = 9.78+j110.23 Ω (Positive sequence impedance)

Z_1_ = 6+j28.5 Ω, Z_2_ = 1.2+j11.5 Ω, Z_3_ = 1.2+j11.5 Ω (Source impedances)

**Figure-1:** Transmission line Network.

Source voltages, G_1_ = 400 kV, G_2_ = 400∠δ1 kV, G_3_ = 400∠δ2 kV.

The distributed parameters per kilometer as follows:

$R_{l0}$ = 0.3215 Ω/km; $X_{l0}$ = 1.1175 Ω/km; $R_{l1}$ = 0.0326 Ω/km; $X_{l1}$ = 0.3674 Ω/km; $C_{1}$ = 12740 μF/km; $C_{0}$ = 7751 μF/km.

The distributed line parameter block set from MATLAB/SIMULINK, 2018a is utilized to build the model for simulation.Where, δ is Load angle in degrees.

The simulation of the test system is conducted at a sampling frequency of 3600 Hz, with 64 samples for one cycle and an operating frequency of 60 Hz. Current signals corresponding to various fault scenarios are gathered at the relaying point and are inputted into the algorithm.

## 3 Basics of 2D- CNN

The basic architecture of CNN with mathematical model is well described in Refs. [35,36,and37]]. The CNN, inspired by biological neural networks, differs from classical neural networks in its ability to learn features directly from raw images, eliminating the need for separate feature extraction techniques [32,33]. CNNs are specifically tailored for processing and analyzing visual data, making them highly effective for tasks like image recognition and classification. They represent a foundational component of computer vision and image processing. A typical 2D CNN architecture comprises alternating convolutional and pooling layers, followed by fully connected layers [32]. This architecture is meticulously designed to hierarchically learn features at varying levels of abstraction, facilitating robust image analysis, as depicted in Fig. 2. Here's a summary of key concepts underlying the theory of 2D CNNs.

**Figure-2:** Basic architecture of 2D- CNN.

### 3.1 Convolutional layers

At the heart of CNNs lies the concept of convolutional layers, which are pivotal in capturing local patterns within input images. These layers utilize small filters or kernels to perform convolution operations across the input image. During this process, each filter is systematically applied, computing the dot product with local regions of the input image at each step. The result is a feature map that highlights the presence of specific features or patterns within the input. By employing multiple filters, CNNs can generate multiple feature maps, each emphasizing different aspects of the input data. The convolution operation is mathematically expressed by equation-1.

(1) $$y_{m}=\sum_{k=0}^{K-1}x_{k}h_{m-k}$$

x: input signal to any CNN layer

h: Kernel convoluted upon the input x

Y: output vector, $[y_{0}\;y_{1}---y_{m}$]

Typically, in CNNs, a non-linear activation function such as ReLU (Rectified Linear Unit) is applied element-wise to the feature maps. This activation function introduces non-linearity, facilitating the learning of complex relationships within the data. The mathematical expression for the ReLU activation function is provided in equation (2).

(2) $$A_{\text{ReLU}}\left(k\right)=\left\{ \begin{array}{c} k\;\text{if}>0\\ 0\;\text{if}\leq 0 \end{array}\right.$$

### 3.2 Pooling layers

Following convolution, pooling layers are frequently employed to down-sample the spatial dimensions of the feature maps. This down-sampling reduces the computational complexity of the network and introduces a degree of translation invariance. Common pooling operations include max pooling and average pooling.

### 3.3 Fully connected layers

Following a series of convolutional and pooling layers, one or more fully connected layers are commonly incorporated into the CNN architecture. These layers establish connections between every neuron in one layer to every neuron in the subsequent layer, enabling the network to discern global patterns and relationships. The final layer in the CNN architecture, termed the classification layer, typically employs the softmax function to make the ultimate prediction. The softmax function's mathematical expression is provided in equation-3.

(3) $$P\left(x_{i}\right)=\frac{e^{x_{i}}}{\sum_{j}e^{x_{j}}}$$

Where, $P\left(x_{i}\right)$ is the probability score of ith output. Finally, the predicted class is chosen as per the highest score among all outputs. In the CNN training process, back propagation and gradient descent techniques are commonly employed. Through these methods, the network iteratively adjusts its weights and biases to minimize a predefined loss function. This loss function typically quantifies the disparity between predicted and true labels. Following training, the predicted class is determined based on the highest probability score among all outputs.

## 4 Continuous wavelet transform (CWT) & scalogram

### 4.1 CWT

The continuous wavelet transform (CWT) is a tool used in signal processing to analyse the frequency content of a signal as it varies over time. Unlike the fourier transform, which provides a single frequency representation for the entire signal, the cwt provides a time-frequency representation, making it particularly useful for non-stationary signals where frequency components change over time. Discrete Wavelet Transform (DWT) is more focused on multi-resolution analysis with specific scaling and shifting of the wavelets. CWT provides a continuous representation of the signal in both time and frequency domains. This continuous representation is particularly useful for capturing the detailed temporal and spectral characteristics of transient fault signals.

The CWT of a signal x(t) is defined as:

(4) $${\text{CWT}}_{m,n}=\int_{-\infty }^{\infty }x\left(t\right)\psi_{m,n}^{*}\left(t\right)\text{dt}$$

Where, $\psi_{m,n}^{*}\left(t\right)=\frac{1}{\sqrt{n}}\psi \left(\frac{t-n}{m}\right)$ is the mother wavelet a function that is localized in both time and frequency.

x(t) is the signal to be transformed.

m is the scale parameter, which is inversely related to frequency.

n is the translation parameter, which shifts the wavelet in time.

The scale parameter m determines the width of the wavelet. Small values of m correspond to high-frequency wavelets (narrow wavelets), while large values of m correspond to low-frequency wavelets (wide wavelets).

### 4.2 Preparation of scalogram images using time-series data and CWT

A scalogram is a visual representation of the magnitude of the CWT coefficients as a function of time and scale. It shows how the frequency content of the signal evolves over time. The step-by-step guide to preparing scalogram images from time-series data, such as fault current data, using the CWT is described below.

a. Obtain Time-Series Data: Start with the time-series data of the fault current. Let's denote this data as i(t).
b. Choose a Mother Wavelet: Select an appropriate mother wavelet ψ(t) based on the characteristics of the signal. Common choices include the Morlet, Morse, Mexican Hat, and Haar wavelets.
c. Compute the CWT: For each combination of scale m and translation n, compute the CWT of the signal i(t).
d. Calculate Magnitudes: Calculate the magnitude of the CWT coefficients $\left|{CWT}_{i\left(m,n\right)}\right|$.
e. Create the Scalogram: Plot the magnitudes of the CWT coefficients as a function of time (translation n) and scale (inverse frequency m). This is typically done using a heatmap or contour plot, where the x-axis represents time, the y-axis represents scale, and the color intensity represents the magnitude of the CWT coefficients.

The x-axis of the scalogram corresponds to time. This allows the representation of how the signal characteristics evolve over time. Fault signals often have distinctive temporal features, such as sudden changes or oscillations, which are captured in the time dimension of the scalogram. The y-axis of the scalogram corresponds to frequency (or scale). This allows the capture of frequency components present in the fault signal at different times. Fault conditions often introduce specific frequency components or harmonics, which are captured in the frequency dimension of the scalogram.

The scalogram provides a joint time-frequency representation, offering a comprehensive view of how the signal's frequency content changes over time.This is particularly useful for non-stationary signals like fault currents, where transient events occur that affect both time and frequency domains. It can be concluded that Scalogram image can capture temporal and frequency domain features.

## 5 Data collection and signal processing

The proposed 2D-CNN deep learning technique for fault detection and classification are discussed in this section. Fig. 3 depicts the summary of proposed approach. The total approach is divided into three steps: Data collection, Data processing, Fault detection and classification.

**Fig. 3:** Summary of proposed 2-D CNN approach.

During data collection stage, faults are created in MATLAB model with different locations and different fault resistances. The different fault types and simulation parameters are mentioned in table-1 for data extraction. The 3-phase current signals are retrieved with specific sampling frequency in per unit (p.u) values as shown in data collection stage of Fig. 3. At the end of this stage data samples are stacked and saved in CPU. There are 11fault classes and one healthy case, all total 12 classes and each class having 300 cases. Total of 12x 300 = 3600 data samples are obtained.

**Table 1:** Fault type and parameters for MATLAB simulation.

Parameters	Fault configurations	Number of cases
Fault type	AG,BG,CG,AB,BC,CA,ABG,BCG,ACG,ABC,ABCG	11
Fault lines(Between Buses)	1-2,1–3,2-3	3
Inception Angle (In degree)	0,30,60,90,120,150,180,210,240,300	10
Fault resistances in ohm	0.01,0.1,1,1.5,5,10,20,30,50,100	10

The second stage, data processing stage is the vital part of the proposed 2D-CNN approach. In this stage continuous wavelet transform(CWT) is applied over fault current signals to convert it into scalogram images as shown in data processing stage of Fig. 3. In this study Morse wavelet is used, the frequency coefficients of each fault data are computed and these coefficients are plotted as scalograms. The MATLAB code used for converting 1-D current signal to 2-D image.The scalogram images of complete data files are saved in CPU. The 2-D scalogram image of fault signals plays an important role in preserving inherent features of raw input data signals and useful for enhancing classification accuracy of fault signals. The scalogram images are saved in CPU as RGB jpeg with 224x224 pixel resolution.

The raw fault current signals and corresponding 2-D scalogram images using CWT are shown in Fig. 4 and (a) shows no-fault current with corresponding scalogram image where Fig. 4(b), (c), 4(d) shows Line to ground fault with 0.001 Ω fault resistance, Line to ground fault with 20 dB noise and Line to ground fault with 1-Ω fault resistance respectively. It is observed from the scalogram images that while adding noises to the signal or changing fault resistance there is a slight change in the images which leads to accurate fault diagnoses of transmission lines. The detailed fault classification is explained in section-6.

**Fig. 4:** Fault Current signals and corresponding 2-D scalogram images.

## 6 Proposed 2D-CNN for fault detection and classification

2D-CNN is a specific kind of CNN that is designed for processing two-dimensional input data such as images. The proposed 2D-CNN implement the most advantageous property of CNN to extract the complex inherent features of transmission line fault signals for detection and classification. The scalogram images of fault currents are used as the input to the 2D-CNN as shown in Fig. 5.

**Fig. 5:** Proposed 2D-CNN for fault classification in Transmission line.

The basic structure of CNN is already discussed in section-3 with diagram. The proposed 2D-CNN structure is different and given in table-2. While designing a 2D-CNN architecture tailored for fault classification tasks. The architecture consisted of multiple convolutional layers followed by pooling layers to automatically extract hierarchical features from the scalogram images. Fully connected layers were then used to perform the final classification. It consists of three convolution layers, two pooling layers and one dense fully connected layer. There is a large similarity amongst fault signals such as LG, LLG and LLLG faults; it is very difficult to accurately distinguish them with their normal features. Convolution and pooling layers are implemented to capture the inherent features from fault images.In this research it is observed that the single convolution and pooling layer is not sufficient to extract all intricated features, so there is a need of multiple convolution and pooling layers to extract accurate features. In the proposed 2D-CNN three convolution and two pooling layers are used after extensive experiments to extract the exact features and improve the fault detection and classification accuracy.

**Table 2:** Structure of proposed 2D-CNN.

Structure of 2D-CNN	Parameters of Layers	Number of Parameters
Convolution Layer-1	Number of Convolution Kernels Size of Convolution Kernel	32 (3,3)
Pooling Layer-1	Max Pooling with window size	(2,2)
Convolution Layer-11	Number of Convolution Kernels Size of Convolution Kernel	64 (3,3)
Pooling Layer-1I	Max Pooling with window size	(2,2)
Convolution Layer-1II	Number of Convolution Kernels Size of Convolution Kernel	64 (3,3)
Dense Fully connected Layer	Number of Neurons	64
Output activation function	Softmax	

The convolution layer plays vital role in the 2D-CNN for accurate feature extraction, at the same time size of the convolution kernel decides the performance of convolution. There is a need of proper kernel size to improve the performance. During fault there is a rapid change in magnitude and phase angle of electrical quantities, if the kernel size is too large, adequate fault features with rapid change in a very short span of time will not be extracted. This may leads to misclassification of actual faults also the large size kernels requires more computational burden which is not acceptable for faster training. In practice it is proven that a (3∗3) convolution kernel can not only extract features accurately but also requires less computational burden [38].Therefore a 3∗3 convolution kernel is designated for proposed research.

## 7 Performance Investigation

### 7.1 Implementation of proposed 2D-CNN

The proposed 2D-CNN model is utilized in python programing using Keras library. MATLAB R2018a is used for modelling and simulation of transmission system to provide time series sampled data of current signal. The sampled current signal is converted to scalogram image using CWT as mentioned in equation-4.All the experiments conducted in a computer having an Intel Core i5 CPU with 8 GB RAM and 64bit operating system.

The total number of classes taken is 12, each class contains 300 images, Total 3600 images are separated into training and testing using 10-fold cross validation. 10-fold cross-validation involves splitting the dataset into 10 equal parts, using 9 parts for training and 1 part for testing, and rotating this process until each part has been used as the test set. This process is repeated 10 times. This methodology ensures that the model's performance is not dependent on a particular train-test split, thus providing a robust assessment of its generalization capabilities. Seventy percentages of total data is used for training and remaining thirty percentages is kept for testing. The epoch and batch size is selected as 10 and 32 respectively. An Adam optimiser is used for training purpose with an initial learning rate of 0.001 and categorical cross entropy as loss function. The key idea behind using Adam is to adaptively adjust the learning rates of each parameter based on the past gradients and past squared gradients. The adaptive nature of Adam allows it to handle different learning rates for each parameter, which can be beneficial when dealing with sparse data or varying importance of features. The process of back propagation and training parameters are updated till the loss function minimized or up to last epoch. The final trained model is obtained to test the performance. The complete flow chart of proposed2D-CNN is given in Fig. 6.

**Fig. 6:** Complete flow chart of proposed 2D-CNN.

The performance indices of proposed classifier: Precision, Recall, F1 score, Specificity and Accuracy are computed as follows,

*Precision*: It measures the model's capacity to correctly identify positive instances out of all the instances it has classified as positive.

(5) $$Precision=\frac{TP}{TP+FP}$$

*Recall*: It quantifies the capability of a model to accurately identify all positive instances in a dataset.

(6) $$Recall=\frac{TP}{TP+FN}$$

*F1 score*: It is harmonic mean of precision and recall, and it yields a balanced measure of model performance that considers both precision and recall.

(7) $$F1-Score=2*\left(\frac{Precision*Recall}{Precision+Recall}\right)$$

*Accuracy*: It measures the overall correctness of a model's predictions.

(8) $$Accuracy=\frac{TP+TN}{TP+TP+FP+FN}$$

The symbols TP,TN,FP and FN are true positive, true negative, false positive and false negative respectively. For training and testing of 2D-CNN multi–class classification Categorical Cross-Entropy loss function is used. The accuracy and loss versus iteration is shown in Fig. 7(a) and Fig.(b) for training and testing. From Fig. 7 it is observed that during the process of training and testing the accuracy is gradually increasing with respect to iterations and reaching at approximately 1 i.e 100 %.Also the loss function decreasing towards zero with respect to iteration. The performance of proposed 2D-CNN model for each class is shown in Table 3, from Table 3. It can be observed from Table 4 that out of 12 classes only line to ground fault (CG) having accuracy of 98.7951 % unless all classes having individual accuracy of 100 %, that leads to an overall accuracy of 99.9074 %.

**Fig. 7:** Accuracy and Loss Curves for Training and testing of 2D CNN.

**Table-3:** Class wise performance of proposed 2D-CNN.

Fault Class	Precision	Recall	Specificity	F1-Score	Accuracy
No-fault	100.00 %	100.00 %	100.00 %	100.00 %	100
AG	100.00 %	100.00 %	100.00 %	100.00 %	100
BG	98.89 %	100.00 %	99.90 %	99.44 %	100
CG	100.00 %	98.80 %	100.00 %	99.85 %	98.7951
AB	100.00 %	100.00 %	100.00 %	99.88 %	100
BC	100.00 %	100.00 %	100.00 %	99.90 %	100
CA	100.00 %	100.00 %	100.00 %	99.91 %	100
ABG	100.00 %	100.00 %	100.00 %	99.93 %	100
BCG	100.00 %	100.00 %	100.00 %	99.94 %	100
ACG	100.00 %	100.00 %	100.00 %	99.95 %	100
ABCG	100.00 %	100.00 %	100.00 %	99.95 %	100
ABC	100.00 %	100.00 %	100.00 %	99.95 %	100
Overall	99.8907 %	99.9074 %	99.9917 %	99.8907 %	99.9074 %

**Table 4:** Class wise performance of proposed 2D-CNN with 20 dB noise.

Fault Class	Precision	Recall	Specificity	F1-Score	Accuracy
No-fault	100	100	100	100	100
AG	98.86	100	99.90	99.43	100
BG	98.89	100	99.90	99.44	100
CG	98.80	98.80	99.90	99.25	98.79
AB	100	100	100	99.88	100
BC	98.91	100	99.90	99.35	100
CA	100	100	100	99.91	100
ABG	100	100	100	99.93	100
BCG	100	100	100	99.93	100
ACG	100	100	100	99.94	100
ABCG	100	97.87	100	99.85	97.87
ABC	100	98.95	100	99.82	98.94
Overall	99.63	99.62	99.96	99.73	99.629

To provide a detailed insight into the classification performance of the proposed model for individual fault types within the testing dataset, a confusion matrix is presented. The confusion matrix, depicted in Fig. 8, showcases the classification outcomes of all fault types, encompassing both accurate and erroneous classifications. Here, the vertical axis represents the true classes, while the horizontal axis signifies the predicted classes. Correctly classified data samples are indicated by the diagonal elements of the confusion matrix, whereas off-diagonal elements denote instances of misclassification. Upon careful examination of the confusion matrix, it is discernible that a minor error occurs in the classification of the line-to-ground fault class (CG), where some data samples of fault type CG are misidentified as BG. However, it is evident that all other classes are correctly classified with a remarkable accuracy rate of 100 %.The summation of all diagonal elements is 1079 and summation of all diagonal elements are 1 i.e one misclassification, it leads to accuracy of (1079/1080) × 100 = 99.9074.Through several trials, an average accuracy of 99.9543 % was attended.

**Fig. 8:** Test confusion matrix of proposed 2D-CNN for fault classification.

To qualitatively illustrate the effectiveness of the proposed 2D-CNN model and assess the separability of features, the nonlinear dimensionality reduction technique t-SNE is utilized to project the data into a two-dimensional space.

The aim is to understand the impact of convolutional layers on fault classification. Visual mappings of features from each convolutional layer are generated using t-SNE, as depicted in Fig. 9. In Fig. 9(a), the distribution of features after the second convolutional layer reveals that the redundancy of fault signals poses challenges in distinguishing between fault types. Subsequently, Fig. 9(b) illustrates that after the third convolutional layer, fault samples from different categories are better organized and clustered the results following the third convolutional layer show that all samples are separated and further clustered into their respective regions, albeit with a minor degree of misclassification.

**Fig. 9:** t-SNE Feature visualisation of convolutional layers.

### 7.2 Performance under noisy environment

Any classifier has to be tested in noise condition for practical implementation. Noise is an integral part of any electrical system; it is also present in electrical power system. The carrier communication lines present in transmission lines produces electromagnetic interference; this is the main source for noise existence in collected data samples. The studied test system is modeled in MATLAB/SIMULINK environment to simulate in noisy condition.In this study an additive white Gaussian noise with 3 different signals to noise ratio(SNR) in dB is added to the collected data samples. The mathematical expression of SNR expressed as

(9) $$\text{SNR}=10*\log\left(\frac{\text{Power}\;\text{of}\;\text{collected}\;\text{signal}}{\text{Power}\;\text{of}\;\text{noise}}\;\right)\;\text{dB}$$

The efficacy of the proposed approach is evaluated with20dB, 30 dB and 40 dB noise The class wise performance with 20 dB is tabulated in table-4 also the confusion matrix under 20 dB noise is depicted in Fig. 10. The Performance comparison of proposed 2D-CNN for fault classification with and without noise are shown in Fig. 11It is observed that in noise free condition accuracy is 99.907 %, in presence of 40 dB and 30 dB noise condition the accuracy of fault classification is reduced to 99.8148 % and 99.72 % whereas it is changing to 99.629 % even under the dense noise of 20 dB.It can be concluded that the proposed 2D-CNN trained with scalogram images detecting and classifying the faults with appreciable higher accuracy in presence of noise condition.

**Fig. 10:** Test confusion matrix of proposed 2D-CNN for fault classification with 20 dB noise.

**Fig. 11:** Performance comparison of proposed 2D-CNN for fault classification with and without noise.

### 7.3 Performance evaluation for high resistance fault

Different researchers has made effort on detecting high resistance faults(HRF) in transmission line [[36], [37], [38]].In most phase-to-ground fault situations, the fault resistances are typically caused by arcs and the grounding of towers, usually ranging between 10 and 20 Ω. However, there are uncommon cases where the resistances are significantly higher. This can happen if a live conductor lands on a high-resistance surface such as sand, rock, cement, or asphalt, or if a tree or branch causes the fault. In these situations, the fault resistances can be much higher, sometimes reaching several hundred ohms. While such faults may not significantly impact power transfer unless a conductor is broken, they pose a serious risk to humans and animals by potentially causing fatal electric shocks. Therefore, it is important to clear high resistance faults even if the resistance is as high as 1000 Ω. In Ref. [39] author presented a suitable method for high resistance fault detection in a two-terminal transmission line based on differential protection with maximum simulation fault resistance of 1kΩ.The proposed study computes differential admittance of pre-fault and fault conditions to identify fault scenario. In Ref. [40] author simulated high resistance fault conditions in a two machine system and faults are simulated over a range of locations, varying from 0 % to 80 % of the line length in 10 % increments, and with different fault resistances set at 5, 50, 100, and 200 Ω and claimed an accuracy of 80 %.Author analyses a real high resistance fault reports of five faults on a 525 kV single-circuit transmission line in south eastern Brazil of 121.4-km line connects the SE Assis Terminal to the SE Londrina Terminal, spanning across São Paulo and Paraná States [41]. Thus it can be concluded that HRF is rare and special case which must be taken care by protection scheme.

To evaluate the effectiveness of the proposed 2D-CNN, data were gathered from various simulation scenarios. Single phase-to-ground faults were initiated at different locations along the line, specifically at 0 %, 25 %, 50 %, 75 %, and 100 % of its length. Fault resistances of 100Ω, 200Ω, 400Ω, 600Ω, 800Ω, 1000Ω, 1200Ω, 1400Ω, 1600Ω, 1800Ω, and 2000Ω were applied at each fault location. Simulations also included scenarios where the line operated with a broken conductor grounded at one or both ends.In total, 300 different high resistance fault (HRF) cases were simulated. Scalogram images were generated from these simulations and incorporated into pre-processed noise-free datasets. The new dataset consisted of 13 classes with dimensions of 13x300. A total of 3900 images were split into training and testing sets using 10-fold cross-validation. Seventy percent of the data was used for training, while the remaining thirty percent was reserved for testing. The chosen epoch and batch size were 10 and 32, respectively. The test confusion matrix of the proposed 2D-CNN for fault classification, utilizing High-Resolution Fault (HRF) data, is depicted in Fig. 12. The model achieves a classification accuracy of 98.46 %. The confusion matrix reveals that HRF instances are sometimes misclassified as AG, BG, CG, and ABG faults. This misclassification likely arises because the HRF simulations were conducted under ground fault conditions. This result demonstrates the efficacy of the 2D-CNN in detecting HRF faults, despite the challenging simulation conditions. It requires more specific research to identify HRF in power system.

**Fig. 12:** Test confusion matrix of proposed 2D-CNN for fault classification with HRF.

### 7.4 Comparative study

A comparative study of the performance of current state-of-the-art techniques involving in fault detection and classification of transmission lines are presented in Table-5. The classification accuracy of these methods are observed both under ideal and noisy conditions with 3 SNR levels of 40 dB, 30 dB and 20 dB respectively. The bar graph of current state-of-art techniques with proposed 2D-CNN are shown in Fig. 13. Although [16,17] have claimed the accuracy of 97.90 % and 84.40 % detection in ideal condition but do not provide any information regarding the performance under noisy condition also used simple ANN. In Ref. [19] author used ANN as classifier and wavelet transform (WT) is utilized for input data processing, obtained an accuracy of 95 % and 97 % for 30 dB and 40 dB noises but ANNs are prone to over fitting, where the model learns to perform well on the training data but fails to generalize to new, unseen data. In Ref. [15] author proposed LSTM as feature extractor and SVM as classifier for two class events and obtained an accuracy of 97.70 % in ideal condition. Though SVM perform well in two class classification, Extending SVMs to handle multiclass classification often requires strategies like one-vs-one or one-vs-all approaches, which can be computationally expensive and lead to suboptimal performance, especially for large numbers of classes. In Ref. [18] author proposed a classification technique for 10 classes using HHT and CNN, obtained an appreciably good accuracy of 99.92 % in ideal data set, author claimed slight less accuracy with 20 dB noise, but actual percentage of accuracy is not clarified. 1D-CNN is proposed in Ref. [24] used 1D-data set of simple double circuit transmission line. Author verified the classifier with 3-sets of different datasets and obtained accuracy of more than 98 %, but the efficacy of the model is not verified in presence of noise.

**Table 5:** Performance comparison of 2D-CNN with other state of art Methods.

Ref. & year	Methods	No. of classes	Data size (Training/Testing)	Considered layers	Classification Accuracy with and without noise			
					ideal	20 dB	30 dB	40 dB
[19]-2017	WT-ANN	10	54336/8066	40	98	–	95	97
[15]-2018	LSTM&SVM	2	4100/1010	5	97.70	–	–	–
[16]-2018	ANN	4	800/150	3	97.90	–	–	–
[17]-2019	ANN	3	208/44	3	84.40	–	–	–
[18]-2019	HTT-CNN	10	1672/1752	6	99.92	–	–	–
[25]-2020	CNN(SET-A)	2	7283 (image)	2	98.27	–	–	–
	CNN(SET-B)	2	1029 (image)	2	98.25	–	–	–
	CNN(SET-C)	2	5145 (image)	2	98.10	–	–	–
[24]-2021	WT-CNN	11	26680/11435	9	99.92	–	–	–
[23]-2022	TSVD-PNN	11	–	–	98.31	99.77	–	–
[26]--2022	CNN-LSTM	11	–	9	98.60	–	–	–
[27]-2023	ELM	11	9909/1102	2	99.18	–	–	–
Proposed	2D-CNN	12	3600/1080 (Scalogram image)		99.9074	99.72	99.8146	99.8146

**Fig. 13:** Bar graph of current state-of-art techniques with proposed 2D-CNN.

1D-CNNs typically operate locally, considering only a fixed-size window of input data at each convolutional layer. This limited receptive field may result in the model being unable to capture long-range dependencies or contextual information that is essential for certain tasks. Author proposed an unsupervised learning Capsule network [23] for fault classification and wavelet decomposed detailed coefficients energy matrix used as input,obtained an accuracy of 98 % with 10 dB SNR. Generating wavelet coefficient-based energy matrices involves complex pre-processing steps, including wavelet decomposition, energy calculation, and potentially additional normalization or scaling. This pre-processing can introduce additional computational overhead and may require careful parameter tuning to ensure optimal performance. In Ref. [22] author obtained an accuracy of 98.31 % using PNN with 20 dB noise also claimed an accuracy of 99.77 % it is to be revivified how the performance of classifier performs better in presence of noise. Again, PNNs typically require storing all training data in memory, as they rely on a non-parametric approach to estimate class conditional probabilities.

Storing large datasets in memory can be computationally expensive and may limit the scalability of PNNs, especially for applications dealing with big data. In Ref. [25] hybrid of CNN and LSTM is proposed for fault identification where CNN is utilized for feature extraction & LSTM is used for training before fully connected layer and obtained an accuracy of 98.60 % but the performance of the model not evaluated in presence of noise. ELM is proposed in Ref. [26]for fault classification and obtained an accuracy of 99.18 % in ideal data set,not evaluated in presence of noise.Though ELMs have fewer hyper parameters to tune compared to traditional neural networks, which can be an advantage for simplicity. However, this lack of tunability can also be a limitation in scenarios where fine-tuning of model parameters is necessary for optimal performance. In complex tasks or datasets with specific characteristics, ELMs may not offer the same level of flexibility as other neural network architectures. The proposed 2D-CNN model has an accuracy of 99.9074 with ideal dataset for 12- class fault classification and performing consistently in presence of noise, as mentioned in table the model having an accuracy of 99.629 %,99.72 % and 99.814 % in 20.30 and 40 dB noises respectively. The performed accuracy demonstrates the efficacy of proposed Scalogram image based 2D-CNN both under ideal and noisy scenarios and performs well as compared to all current state-of-art fault detection techniques.

## 8 Conclusion

In conclusion, this study introduces a robust and effective methodology for fault detection and classification in transmission lines, leveraging the power of 2D-CNN. By converting fault signals into scalogram image using CWT, the proposed approach captures intricate spatial and temporal patterns, enhancing the discrimination of various fault types. The comprehensive evaluation of the model against transmission line data sets demonstrates its superior performance in terms of accuracy and robustness. The interpretability analysis of the trained 2D-CNN using t-sne graphs after each convolution provides valuable insights into the features influencing fault detection and classification. The proposed 2D-CNN model has an accuracy of 99.9074 with ideal dataset for 12- class fault classification and performing consistently in presence of noise, especially under challenging conditions like high resistance faults and noisy environments as mentioned in table the model having an accuracy of 99.629 %,99.72 % and 99.814 % in 20,30 and 40 dB noises respectively.The scalability and efficiency of the proposed methodology make it well-suited for real-time fault analysis in large-scale power transmission systems. As an advanced tool for fault detection, the 2D-CNN model holds great potential for enhancing the resilience of electrical grids by enabling swift and accurate responses to transmission line disturbances. The demonstrated capabilities of the 2D-CNN model with scalogram fault images out performs the current state-of-art techniques and underscore its relevance for future advancements in fault detection technology.

## Future scope

Future research will focus on studying the impact of high penetration of renewable energy sources, such as wind and solar, on fault characteristics and detection methods. The variability and intermittency associated with renewable energy sources introduce unique challenges that can affect traditional fault detection and classification approaches. Additionally, the influence of **power swings** caused by large system disturbances needs to be explored. These swings can mimic fault conditions and impact the proposed algorithm's accuracy in distinguishing between swings and genuine faults. Improving the algorithm's ability to differentiate between these phenomena is essential for maintaining reliability during dynamic system conditions. The impact of **FACTS devices** (e.g., SVC, STATCOM, TCSC) on fault detection and classification remains a significant area of future research [42]. FACTS devices alter power flow and impedance characteristics, which can influence fault detection accuracy. Developing dynamic models of FACTS-compensated transmission lines will enable more precise simulation and analysis of fault scenarios, providing deeper insights into system behaviour and aiding in the development of robust detection methods. Lastly, implementing **data-driven approaches** that utilize real-time data from smart grid sensors and IoT devices can greatly enhance fault detection systems. This real-time data can be used to train and validate fault detection models, making them more adaptive and responsive to actual operating conditions.

## CRediT authorship contribution statement

**Pravati Nayak:** Resources, Project administration, Methodology. **Shitya Ranjan Das:** Visualization, Validation, Software. **Ranjan K. Mallick:** Writing – original draft, Visualization, Supervision. **Sairam Mishra:** Writing – original draft, Visualization, Resources. **Ahmed Althobaiti:** Resources, Project administration, Methodology. **Alsharef Mohammad:** Writing – original draft, Validation, Project administration. **Flah Aymen:** Writing – review & editing, Writing – original draft, Supervision, Investigation, Funding acquisition.

## Declaration of competing interest

The authors declare that they have no known competing financial interests or personal relationships that could have appeared to influence the work reported in this paper.

## References

[1] Paithankar Y.G., Bhide S.R. (2010).

[2] Bahmanyar A. (2017). A comparison framework for distribution system outage and fault location methods. Elec. Power Syst. Res..

[3] Bhatnagar M., Yadav A. (2020). 2020 5th IEEE International Conference on Recent Advances and Innovations in Engineering (ICRAIE).

[4] Jana S., De A. (2017). 2017 IEEE Calcutta Conference (CALCON).

[5] Chen K., Huang C., He J. (2016). Fault detection, classification and location for transmission lines and distribution systems: a review on the methods. High Volt..

[6] Jamehbozorg A., Shahrtash S.M. (2010). A decision-tree-based method for fault classification in single-circuit transmission lines. IEEE Trans. Power Deliv..

[7] Ray P., Mishra D.P. (2016). Support vector machine based fault classification and location of a long transmission line. Engineering science and technology, an international journal.

[8] Taheri M.M., Seyedi H., Mohammadi‐ivatloo B. (2017). DT‐based relaying scheme for fault classification in transmission lines using MODP. IET Generation, Transmission & Distribution.

[9] Cervantes J., Garcia-Lamont F., Rodríguez-Mazahua L., Lopez A. (2020). A comprehensive survey on support vector machine classification: applications, challenges and trends. Neurocomputing.

[10] Zhang P., Shu S., Zhou M. (2018). An online fault detection model and strategies based on SVM-grid in clouds. IEEE/CAA Journal of Automatica Sinica.

[11] Fonseca Gabriel A. (2022). Fault classification in transmission lines using random forest and notch filter. Journal of Control, Automation and Electrical Systems.

[12] Mohanty Subodh Kumar, Karn Anshudip, Banerjee Shobhan (2020). 2020 IEEE International Conference on Power Electronics, Smart Grid and Renewable Energy (PESGRE2020).

[13] Sheykhmousa Mohammadreza (2020). Support vector machine versus random forest for remote sensing image classification: a meta-analysis and systematic review. IEEE J. Sel. Top. Appl. Earth Obs. Rem. Sens..

[14] Li Zewen (2021). A survey of convolutional neural networks: analysis, applications, and prospects. IEEE Transact. Neural Networks Learn. Syst..

[15] Zhang Senlin (2017). Data-based line trip fault prediction in power systems using LSTM networks and SVM. IEEE Access.

[16] Padhy Santosh K. (2018). 2018 International Conference on Information Technology (ICIT).

[17] Fahim Shahriar Rahman (2019). 2019 IEEE International Conference on Power, Electrical, and Electronics and Industrial Applications (PEEIACON).

[18] Guo Mou-Fa, Yang Nien-Che, Chen Wei-Fan (2019). Deep-learning-based fault classification using Hilbert–Huang transform and convolutional neural network in power distribution systems. IEEE Sensor. J..

[19] Abdullah Ahmad (2017). Ultrafast transmission line fault detection using a DWT-based ANN. IEEE Trans. Ind. Appl..

[20] Mukherjee Alok (2021). Probabilistic neural network-aided fast classification of transmission line faults using differencing of current signal. J. Inst. Eng.: Series.

[21] Chen Yann Qi, Fink Olga, Sansavini Giovanni (2017). Combined fault location and classification for power transmission lines fault diagnosis with integrated feature extraction. IEEE Trans. Ind. Electron..

[22] Mishra Praveen Kumar, Yadav Anamika (2024). E-Prime-Advances in Electrical Engineering, Electronics and Energy.

[23] Rajesh P. (2022). Optimally detecting and classifying the transmission line fault in power system using hybrid technique. ISA Trans..

[24] Fahim Shahriar Rahman (2021). A deep learning based intelligent approach in detection and classification of transmission line faults. Int. J. Electr. Power Energy Syst..

[25] Liu Yiqing, Zhu Yiming, Wu Kai (2020). CNN-based fault phase identification method of double circuit transmission lines. Elec. Power Compon. Syst..

[26] Moradzadeh Arash (2022). Hybrid CNN-LSTM approaches for identification of type and locations of transmission line faults. Int. J. Electr. Power Energy Syst..

[27] Goni Md Omaer Faruq (2023). Fast and accurate fault detection and classification in transmission lines using extreme learning machine. e-Prime-Advances in Electrical Engineering, Electronics and Energy.

[28] Khodayar Mahdi (2020). Deep learning in power systems research: a review. CSEE Journal of Power and Energy Systems.

[29] Biswas Sauvik (2023). An intelligent fault detection and classification technique based on variational mode decomposition-CNN for transmission lines installed with UPFC and wind farm. Elec. Power Syst. Res..

[30] Biswas Sauvik (2023). IEEE Journal of Emerging and Selected Topics in Industrial Electronics.

[31] Li Wenting (2019). Real-time faulted line localization and PMU placement in power systems through convolutional neural networks. IEEE Trans. Power Syst..

[32] Mujtaba Ghulam, Malik Adeel, Ryu Eun-Seok (2022). LTC-SUM: lightweight client-driven personalized video summarization framework using 2D CNN. IEEE Access.

[33] Yin Rui (2021). IAV-CNN: a 2D convolutional neural network model to predict antigenic variants of influenza A virus. IEEE ACM Trans. Comput. Biol. Bioinf.

[34] Samantaray S.R., Kamwa I., Joos Geza (2011). Decision tree based fault detection and classification in distance relaying. International Journ Engineering Intelligent Systems Electrical Engineering Communications.

[35] Taye Mohammad Mustafa (2023). Theoretical understanding of convolutional neural network: concepts, architectures, applications, future directions. Computation.

[36] Indolia Sakshi (2018). Conceptual understanding of convolutional neural network-a deep learning approach. Procedia computer science.

[37] Kuo C-C. Jay (2016). Understanding convolutional neural networks with a mathematical model. J. Vis. Commun. Image Represent..

[38] Hammad Issam, El-Sankary Kamal (2018). Impact of approximate multipliers on VGG deep learning network. IEEE Access.

[39] Łukowicz M. (2010).

[40] Makwana Vijay H., Bhalja Bhavesh R. (2012). A new digital distance relaying scheme for compensation of high-resistance faults on transmission line. IEEE Trans. Power Deliv..

[41] Maezono Paulo Koiti (2009). 2009 62nd Annual Conference for Protective Relay Engineers.

[42] Biswas Sauvik, Ketan Panigrahi Bijaya (2024). An improved fault detection and phase identification for collector system of DFIG-wind farms using least square transient detector coefficient. Elec. Power Syst. Res..

